# Quality control material for the detection of somatic mutations in fixed clinical specimens by next-generation sequencing

**DOI:** 10.1186/s13000-015-0403-0

**Published:** 2015-09-17

**Authors:** Catherine I. Dumur, Jorge A. Almenara, Celeste N. Powers, Andrea Ferreira-Gonzalez

**Affiliations:** Department of Pathology, Virginia Commonwealth University, Clinical Support Center, Room 247, 403 North 13th Street, Richmond, VA 23298 USA

## Abstract

**Background:**

Targeted next generation sequencing (NGS) technology to assess the mutational status of multiple genes on formalin-fixed, paraffin embedded (FFPE) tumors is rapidly being adopted in clinical settings, where quality control (QC) practices are required. Establishing reliable FFPE QC materials for NGS can be challenging and/or expensive. Here, we established a reliable and cost-effective FFPE QC material for routine utilization in the Ion AmpliSeq™ Cancer Hotspot Panel v2 (CHP2) assay.

**Methods:**

The performance characteristics of the CHP2 assay were determined by sequencing various cell line mixtures and 55 different FFPE tumors on the Ion Torrent PGM platform. A FFPE QC material was prepared from a mixture of cell lines derived from different cancers, comprising single nucleotide variants and small deletions on actionable genes at different allelic frequencies.

**Results:**

The CHP2 assay performed with high precision and sensitivity when custom variant calling pipeline parameters where established. In addition, all expected somatic variants in the QC material were consistently called at variant frequencies ranging from 9.1 % (CV = 11.1 %) to 37.9 % (CV = 2.8 %).

**Conclusions:**

The availability of a reliable and cost-effective QC material is instrumental in assessing the performance of this or any targeted NGS assay that detects somatic variants in fixed solid tumor specimens.

## Background

The numerous cancer genome characterization efforts that have emerged in the past years [1–3] have promoted the development of targeted cancer therapeutics [4], including single or combined inhibitory agents [5], which reportedly are beneficial to individuals who have tumors harboring specific somatic mutations in genes encoding for proteins involved in cell growth, proliferation, and survival signaling pathways [6–9]. Thus, molecular testing to identify such mutations in clinical specimens to assess patient eligibility for targeted therapies has become standard practice in the management of oncology patients.

The recent technological advances in next-generation sequencing (NGS) and the applications in the field of oncology are revolutionizing clinical testing for personalized treatment decisions for oncology patients [10]; as well as the translational research field, where somatic variant findings may enhance the development of novel targeted cancer therapeutics, which could benefit individuals with tumors harboring such mutations. A variety of different NGS-based assays have been developed for mutation identification that have the ability to detect all mutation types, including single nucleotide variants (SNVs), copy number variants (CNVs), insertion/deletions (Indels) and translocations, in many samples and many genomic regions simultaneously, while providing a digital readout of mutation frequencies.

The advent of NGS benchtop sequencers has allowed the rapid adoption of molecular testing for somatic mutations in clinical settings [11–13]. Thus, amplifying discrete or targeted regions of the genome has allowed for the development of panels of “amplicon sequencing.” As an example, the Ion AmpliSeq™ Cancer Hotspot Panel v2 (Life Technologies, Carlsbad, CA), which targets 207 exonic regions across 50 cancer-relevant genes, is producing robust results starting from 1 to 10 ng of DNA isolated from formalin-fixed, paraffin embedded (FFPE) specimens [14]. Such an assay can yield up to 1 gigabyte (Gb) of DNA sequence in the Ion Torrent Personal Genome Machine™ (PGM), depending on the chip used to run the sequencing reaction, in short DNA fragments. Similarly, the TruSeq Amplicon - Cancer Panel (Illumina, Inc., San Diego, CA), assay allows the sequencing of mutational hotspots located in 212 exonic regions corresponding to 48 cancer-related genes on the Illumina MiSeq, from 250 ng of DNA sample. These NGS platforms provide the benefit of targeting multiple genomic regions in a single reaction, thus lowering the cost of the assay and allowing for testing multiple genes in small samples.

However, the performance characteristics of NGS-based clinical assays needs to be assessed during the assay validation process, and ensured during routine clinical runs [15]. One of the remaining challenges for NGS-based clinical assays is the availability of robust, cost effective, reference or quality control (QC) material. Access to such material is crucial to be able to generate confident NGS results, while managing potential workflow variability from sample extraction to sequencing, data analysis pipeline and variant calling.

In this study we describe the analytical and clinical validation of a 50-gene NGS assay, the Ion AmpliSeq™ Cancer Hotspot Panel v2 (CHP2), performed on the Ion Torrent PGM, for clinical testing, as well as the development of a robust, and relatively low cost, QC material to assess performance characteristics during routine clinical runs.

## Materials and methods

### Cell lines

DNA isolated from fresh-frozen, as well as from formalin-fixed, paraffin-embedded (FFPE) cell pellets from melanoma (SK-MEL28), pancreatic (MIA-PaCa-2), colon (HCT116), and lung (H1975) cancer cell lines was used. All the cell lines were obtained from American Type Culture Collection (ATCC-http://www.atcc.org, Manassas, VA). Each individual cell line DNA sample was sequenced alone or combined with others in different proportions, resulting in various sample mixes harboring different mutations, at different frequencies.

### Tissue specimens

Fifty five de-identified archival DNA samples isolated from FFPE tissue blocks containing greater than 40 % neoplastic cells (43 non-small cell lung carcinoma (NSCLC), 4 colorectal cancer, and 8 melanoma cases) with known mutational status for the *KRAS*, *EGFR* and *BRAF* (including 25 Negative and 30 Positive for mutations in at least one of these three genes) were used for the clinical validation of the CHP2 assay. These DNA samples had previously been isolated from tumor-enriched samples by manual Microdissection, when indicated by a pathologist.

### Single gene mutation assays

*KRAS* mutations in codons 12 and 13 were detected by Sanger sequencing, preceded by a Co-amplification at Lower Denaturation-temperature PCR (COLD-PCR) [16] step for allele enrichment, whereas *EGFR* mutations in exons 18 to 21 were detected by Scorpion primer-probes and Amplification Refractory Mutation Screening (ARMS®) [17] technology using the real-time PCR-based EGFR RGQ PCR assay (Qiagen, Valencia, CA) according to the manufacturer’s recommendations. *BRAF* mutations in the V600 codon, as well as specific *SMAD4* and *RET* variants, were detected by multiplex allele-specific PCR (AS-PCR) reactions that co-amplify the variant sequence and an upstream conserved sequence, where amplicons were detected by capillary electrophoresis using Lab-on-a-Chip technology. The primers used for the multiplex AS-PCR amplification for *BRAF*, *SMAD4* and *RET* specific variants are listed in Table 1, along with the resulting amplicon sizes.

**Table 1:** ASPCR Primers

Amplicon Name	Primer Sequence (5'-3')	Amplicon Size (bp)
BRAF_conserved	BRAF-F1: TGCTTGCTCTGATAGGA	241
	BRAF_R: CTAGTAACTCAGCAGCA	
BRAF_V600E	BRAF-F2: TGGTCTAGCTACAGA	141
	BRAF_R: CTAGTAACTCAGCAGCA	
SMAD4_conserved	SMAD4_F1: TTGTCTTTTCTTTAGGGC	286
	SMAD4_R: AAGATAGTTCTTTTCTTTTGG	
SMAD4_48586344_C > T	SMD4_F2: ATTTAGTGGTGATTGAAAT	181
	SMAD4_R: AAGATAGTTCTTTTCTTTTGG	
RET_conserved	RET_F1: GTGCTATTTTTCCTCACA	268
	RET_R: AGGGCTATAAAAAGCTTAG	
RET_43615612_A > G	RET_F2: GCTTGTCCCGG	176
	RET_R: AGGGCTATAAAAAGCTTAG	

### DNA isolation

All tissue H&E stained slides were reviewed by a pathologist who assessed percent tumor content and delineated the tumor area for manual microdissection, if needed. Ten-micron unstained FFPE slides were then manually dissected, when indicated, and DNA was extracted using the DNA mini kit as described by the manufacturer (Qiagen, Germantown, MD). The same DNA extraction method was used for the fresh-frozen and FFPE cell line pellets and from specimens subjected to laser capture microdissection (LCM). Double-stranded DNA (dsDNA) yield and concentration was assessed by fluorometry on the Qubit® 2.0 instrument (Life Technologies, Carlsbad, CA)

### Library preparation

The Ion AmpliSeq™ Cancer Hotspot Panel v2 (CHP2) was used to generate 207 amplicons covering over 2,800 hotspots, indexed in the COSMIC database, in 50 cancer-related genes, from 1 to 10 ng of dsDNA for each sample, using additional PCR cycles for the lowest dsDNA concentrations. The multiplexed amplicons were then used to generate barcoded libraries using the Ion AmpliSeq™ Library Kit 2.0 and the Ion Xpress™ barcoded adapters (Life Technologies, Carlsbad, CA). Amplified libraries were quantitated following the manufacturer's recommendations. Barcoded libraries were combined to a final concentration of 7 pM, to achieve optimal yield of clonal templated Ion Sphere™ Particles (ISPs), for emulsion PCR (emPCR) and further ISP enrichment following the manufacturer's recommendations. Sequencing was performed on 316™ chips run on the Ion Torrent PGM and analyzed with the Torrent Suite v4.0.2 Software. The February 2009 assembly of the human genome (hg19, GRCh37 Genome Reference Consortium Human Reference 37) was used as a reference.

### Determining the Limit of Detection (LoD)

DNA mixes from the four fresh-frozen cell line pellets used in this study were further diluted in DNA isolated from a de-identified normal snap-frozen human placenta to achieve several different variants at different frequencies 39 variants in 24 genes. In addition, DNA isolated from FFPE cell line pellets was combined in different proportions to achieve 37 variants at different frequencies in 23 genes.

### Analytical performance evaluation

Robustness, repeatability and reproducibility were assessed by preparing multiple libraries from the LoD sample mixtures and running them in different 316™ chips. Accuracy was evaluated by comparing variant frequencies obtained from individual cell lines with the results obtained by the Genomics and Bioinformatics Group (GBG) from NCI, by querying the CellMiner database [18]. In addition, libraries from the 55 patient samples and from the well-characterized reference DNA sample NA12878 from the HapMap project [19] were sequenced and compared to single gene mutation assay results to further assess the accuracy of the CHP2 assay.

### Data analysis pipeline

The sequencing data generated by the Ion Torrent PGM was stored and analyzed in the Linux-based Server, based on Ubuntu operating system, connected to the instrument. The file types created during sequencing included: raw image acquisition . DAT files; base-calling, resulting in an unmapped BAM format file; and alignment to the reference genome using the TMAP aligner algorithm, with the output being a BAM file. Output BAM files, along with target regions BED files, were used for variant identification by the *VariantCaller* plugin. Visualization of the raw alignments was assessed using the Broad's Integrative Genomics Viewer (IGV 2.3.11) [20].

### Variant calling

The Torrent *VariantCaller* (TVC) plugin was used to identify and evaluate variants. The CHP2 assay was validated with the TVC 4.0 version of the plugin. The TVC 4.0 is designed to call SNVs, multi-nucleotide variants (MNVs), insertions (INS), and deletions (DEL). The analysis pipeline uses FreeBayes, based on user-modifiable parameters, such as coverage, quality, strand bias, and homopolymer length, among others, to discover candidate variant locations, which are subsequently scored using adaptive signal model and filtered. FreeBayes [21] is a haplotype-based variant detector that runs in a Bayesian statistical framework, which is capable of modeling multiallelic loci in sets of individuals with non-uniform copy number. Afterwards, a second module performs assembly of reads to detect long INS and/or DEL (Indels). A set of seven barcoded FFPE cell line mix samples with known variant frequencies were used to establish cutoff values for critical TVC parameters to achieve enough stringency (fewer false positives), while maintaining high sensitivity (fewer false negatives) in the variant calling process. For each critical parameter, z-scores of normally distributed data were calculated to establish cutoff values to be used the custom TVC plugin parameters, which were recorded in a JSON text format. We used the Shapiro-Wilk normality test [22] to assess the normality of the critical parameters distribution.

### Quality Control (QC) material

QC material was prepared by growing the four cell lines in individual T-75 flasks up to right before they reach confluence. Then, cells were scrapped off each flask and pooled together in PBS. This cell mixture was centrifuged for 10 min at 1800 rpm and the supernatant was decanted. The cell pellet was then resuspended in 500 μL of normal human plasma. Fifty μL of thrombin solution (Siemens Healthcare Diagnostics Inc., Tarrytown, NY) were added to the cell pellet/plasma mixture to allow a clot to form. The cell-containing clot was further fixed in formalin for 9 h (typical fixation time for human tissues in our laboratory), and embedded in paraffin following the routine processing for fine-needle aspiration (FNA) cell pellets. DNA was isolated from a single 10-μm section from the cell mixture block, in parallel with patient samples in each batch of samples, and was sequenced in every run as an individual barcoded library with six more libraries from patient samples in 316™ chips. For the QC material, variants and their frequencies were first assessed by sequencing this material in 10 consecutive runs on the Ion Torrent PGM to establish the performance characteristics (i.e., Mean, +2SD, +3SD, etc.…) of each variant. After implementing this quality control material in clinical runs, the same variants and their frequencies were monitored over time using Levey-Jennings control charts.

## Results

### Analytical performance characteristics

From the DNA dilution experiments, where DNA isolated from the four fresh-frozen cell line pellets was further diluted in DNA isolated from a de-identified normal human placenta, we were able to detect the variants, both SNV and DEL, at the frequencies listed in Table 2. Since variants with frequencies near 3 % were called only 90 % of the time, we established the limit of detection (LoD) at 4 % mutant DNA in the context of normal DNA for fresh-frozen samples, which were detected 100 % of the time when barcoding up to seven samples with an average coverage of near 2000X per sample (Fig. 1). In addition, the same samples run using different barcodes within the same chip, or the same barcode on different chips, showed excellent correlations indicating high repeatability and reproducibility, respectively (Fig. 2).

**Table 2:** Variants identified in DNA isolated from frozen cell line mixes

				Cell Line / Sample Name	HCT116	MiaPaCa-2	H1975	SK-MEL-28	4-Cell Line Mix		Human Placenta	4-Cell Line Mix (Dil 1:2)		4-Cell Line Mix (Dil 1:3)	
Gene Symbol	hg19 Coordinates	Variant Type	Variant	Freq. (%)	Found	Found	Found	Found	Expected	Found	Found	Expected	Found	Expected	Found
*ABL1*	133738370	SNV	G		52.4	N.A.	N.A.	N.A.	13.1	12.6 ± 0.5	N.A.	6.1	6.3 ± 0.2	4.1	4.4 ± 0.5
*APC*	112175770	SNV	A		98.1	74.4	51.7	88.5	78.1	80.0 ± 0.9	2.1	40.7	40.8 ± 0.9	27.8	29.4 ± 0.8
*ATM*	108138003	SNV	C		N.A.	N.A.	N.A.	N.A.	N.A.	N.A.	55.8	27.9	32.1 ± 0.2	37.2	40.6 ± 0.4
*BRAF*	140453136	SNV	A		N.A.	N.A.	N.A.	99.3	24.8	21.7 ± 4.0	N.A.	12.3	13.7 ± 0.2	8.2	9.6 ± 0.2
*CDKN2A*	21971153	SNV	T		N.A.	N.A.	96.4	N.A.	24.1	35.7 ± 2.6	N.A.	16.9	10.4 ± 1.1	11.3	8.4 ± 0.9
*CSF1R*	149433596	SNV	C		99.6	99.3	100.0	N.A.	74.7	58.6 ± 4.5	90.5	72.9	68.8 ± 0.6	78.8	80.5 ± 1.2
*CSF1R*	149433597	SNV	T		99.6	99.1	100.0	N.A.	74.7	62.3 ± 9.8	93.2	74.3	76.9 ± 0.7	80.6	85.7 ± 0.8
*CTNNB1*	41266134	DEL	CTT		50.2	N.A.	N.A.	N.A.	12.5	10.7 ± 1.8	N.A.	4.7	4.8 ± 0.6	3.2	3.1^a^ ± 0.1
*EGFR*	55242487	SNV	T		N.A.	N.A.	N.A.	99.3	24.8	22.8 ± 2.6	N.A.	12.3	13.4 ± 0.1	8.2	8.0 ± 0.6
*EGFR*	55249063	SNV	A		100.0	23.2	70.6	100.0	73.4	75.3 ± 1.7	97.6	85.9	84.4 ± 0.7	89.8	90.1 ± 0.3
*EGFR*	55249071	SNV	T		N.A.	N.A.	70.7	N.A.	17.7	27.1 ± 2.5	N.A.	12.7	13.6 ± 1.1	8.4	8.9 ± 1.2
*EGFR*	55259515	SNV	G		N.A.	N.A.	56.7	N.A.	14.2	17.8 ± 0.7	N.A.	9.2	8.8 ± 1.3	6.1	6.4 ± 0.5
*ERBB4*	212812097	SNV	G		100.0	N.A.	75.9	N.A.	44.0	54.0 ± 0.2	62.9	58.4	46.8 ± 1.6	59.9	59.0 ± 2.3
*FGFR3*	1807894	SNV	A		100.0	100.0	99.6	100.0	99.9	99.6 ± 0.2	100.0	99.9	99.9 ± 0.1	99.9	99.8 ± 0.1
*FLT3*	28602367	SNV	A		46.9	N.A.	N.A.	N.A.	11.7	15.4 ± 3.2	N.A.	8.8	7.0 ± 0.3	5.9	6.4 ± 0.8
*FLT3*	28610183	SNV	C		100.0	66.5	99.6	69.2	83.8	80.9 ± 1.1	100.0	90.9	90.8 ± 0.1	93.9	93.4 ± 0.5
*HRAS*	534242	SNV	C		99.5	61.9	40.4	46.9	62.2	67.6 ± 1.1	2.6	34.7	32.0 ± 0.2	24.0	21.5 ± 1.2
*KDR*	55946354	SNV	A		48.5	N.A.	N.A.	N.A.	12.1	15.9 ± 1.0	51.3	33.3	34.5 ± 1.1	39.3	41.0 ± 1.1
*KDR*	55972974	SNV	T		52.6	N.A.	N.A.	N.A.	13.1	13.2 ± 4.3	N.A.	8.1	7.3 ± 0.5	5.4	5.1 ± 0.1
*KRAS*	25398281	SNV	A		46.4	N.A.	N.A.	N.A.	11.6	11.3 ± 0.7	N.A.	5.9	6.2 ± 0.4	3.9	4.2 ± 0.1
*KRAS*	25398285	SNV	T		N.A.	99.9	N.A.	N.A.	25.0	24.7 ± 1.2	N.A.	12.8	13.7 ± 0.5	8.5	9.5 ± 0.1
*MET*	116339672	SNV	T		N.A.	72.9	N.A.	N.A.	18.2	15.3 ± 2.0	N.A.	6.9	7.9 ± 0.0	4.6	4.8 ± 0.1
*NOTCH1*	139390822	SNV	G		N.A.	100.0	N.A.	N.A.	25.0	22.5 ± 0.3	N.A.	11.1	9.3 ± 0.2	7.4	7.1 ± 0.1
*PDGFRA*	55141055	SNV	G		99.7	100.0	99.7	100.0	99.8	99.9 ± 0.2	99.9	99.8	99.9 ± 0.1	99.8	100.0 ± 0.1
*PDGFRA*	55152040	SNV	T		N.A.	N.A.	50.8	N.A.	12.7	11.8 ± 2.8	3.8	8.8	7.5 ± 0.1	7.1	6.0 ± 0.7
*PIK3CA*	178917005	SNV	G		N.A.	N.A.	100.0	N.A.	25.0	28.6 ± 7.6	N.A.	11.6	13.9 ± 0.1	7.8	10.2 ± 0.6
*PIK3CA*	178927410	SNV	G		N.A.	N.A.	45.1	N.A.	11.3	10.7 ± 1.2	N.A.	5.8	5.9 ± 0.2	3.9	4.0 ± 0.2
*PIK3CA*	178952085	SNV	G		47.7	N.A.	N.A.	N.A.	11.9	11.3 ± 2.3	N.A.	4.9	6.4 ± 0.4	3.2	3.9^a^ ± 0.1
*PTEN*	89711881	SNV	G		N.A.	N.A.	N.A.	99.3	24.8	24.3 ± 1.0	N.A.	11.8	9.5 ± 0.8	7.9	8.4 ± 0.6
*RET*	43613843	SNV	T		100.0	65.8	100.0	N.A.	66.4	70.8 ± 2.1	100.0	86.1	86.8 ± 0.6	90.7	91.3 ± 0.5
*RET*	43615612	SNV	G		45.2	N.A.	N.A.	N.A.	11.3	15.1 ± 0.3	N.A.	7.4	7.2 ± 0.3	5.0	2.9 ± 0.5
*RET*	43615633	SNV	G		N.A.	64.5	N.A.	N.A.	16.1	14.1 ± 0.0	N.A.	7.1	7.6 ± 0.5	4.7	3.7 ± 1.1
*SMAD4*	48586344	SNV	T		47.6	N.A.	N.A.	N.A.	11.9	17.2 ± 1.4	N.A.	8.1	6.5 ± 0.2	5.4	4.9 ± 0.2
*SMARCB1*	24176287	SNV	A		50.7	N.A.	40.8	N.A.	22.9	22.0 ± 2.3	N.A.	11.8	14.6 ± 0.1	7.9	10.7 ± 0.4
*SMO*	128846374	SNV	A		52.6	N.A.	N.A.	N.A.	13.1	10.5 ± 1.5	N.A.	5.8	7.8 ± 2.0	3.9	4.4 ± 0.2
*TP53*	7577025	SNV	T		N.A.	N.A.	N.A.	N.A.	N.A.	N.A.	79.0	39.5	29.1 ± 1.5	52.6	41.4 ± 1.1
*TP53*	7577120	SNV	A		N.A.	N.A.	99.9	N.A.	25.0	31.6 ± 2.6	N.A.	16.7	20.8 ± 0.8	11.1	16.0 ± 0.1
*TP53*	7577539	SNV	T		N.A.	99.5	N.A.	N.A.	24.9	18.8 ± 0.7	N.A.	9.6	11.3 ± 0.1	6.4	9.1 ± 0.1
*TP53*	7579472	SNV	G		94.2	N.A.	94.2	N.A.	47.1	63.6 ± 8.9	20.4	45.1	54.3 ± 2.3	36.9	42.7 ± 1.7

Freq. Frequency; N.A., Not Applicable; a, these variants were called 90 % of the time

**Fig. 1:** Limit of Detection (LoD) and linearity of the CHP2 assay. DNA isolated from four fresh-frozen cell line pellets was further diluted in DNA isolated from a de-identified normal human placenta. Variants were identified at the expected frequencies, down to 3 % mutant DNA in the context of normal DNA for fresh-frozen samples, when barcoding up to 7 samples. Pearson correlation is shown. Dotted line denotes the equality line

**Fig. 2:** Precision of the CHP2 assay. A representative sample run using different barcodes on the same chip to assess repeatability (**a**), or the same barcode on different chips to assess reproducibility (**b**). Pearson correlation is shown. Dotted line denotes the equality line

From the DNA dilution experiments, where DNA isolated from different FFPE cell line pellets was mixed in different proportions, we were able to detect the variants, at different frequencies (Table 3) without affecting the LoD found with DNA isolated from fresh-frozen specimens, when barcoding up to seven samples with an average coverage of near 1300X per sample.

**Table 3:** Variants identified in DNA isolated from FFPE cell line mixes

				Cell Line/Sample Name	HCT116	MiaPaCa-2	H1975	SK-MEL-28	4-Cell Line Mix		H1975 Dil in MiaPaCa-2 (1:14)	
Gene Symbol	hg19 Coordinates	Variant Type	Variant	Frequency (%)	Found	Found	Found	Found	Expected	Found	Expected	Found
*ABL1*	133738370	SNV	G		37.0	N.A.	N.A.	N.A.	9.3	12.4 ± 2.6	0.0	N.A.
*APC*	112175770	SNV	A		98.0	72.7	36.5	91.3	74.6	78.4 ± 1.2	70.2	65.4 ± 1.4
*BRAF*	140453136	SNV	A		N.A.	N.A.	N.A.	100.0	25.0	21.1 ± 2.5	0.0	N.A.
*CDKN2A*	21971153	SNV	T		N.A.	N.A.	98.8	N.A.	24.7	17.9 ± 0.6	100.0^a^	98.6 ± 0.9
*CSF1R*	149433596	SNV	C		100.0	100.0	100.0	N.A.	75.0	61.4 ± 2.6	100.0	99.9 ± 0.2
*CSF1R*	149433597	SNV	T		95.7	96.1	97.2	N.A.	72.3	58.0 ± 3.7	96.2	97.2 ± 0.9
*CTNNB1*	41266134	DEL	CTT		44.9	N.A.	N.A.	N.A.	11.2	12.9 ± 1.6	0.0	N.A.
*EGFR*	55242487	SNV	T		N.A.	N.A.	N.A.	100.0	25.0	20.9 ± 0.1	0.0	N.A.
*EGFR*	55249063	SNV	A		100.0	35.6	75.3	100.0	77.7	74.0 ± 3.2	38.4	48.1 ± 0.6
*EGFR*	55249071	SNV	T		N.A.	N.A.	74.8	N.A.	18.7	17.9 ± 0.9	5.2	30.4 ± 1.3
*EGFR*	55259515	SNV	G		N.A.	N.A.	71.7	N.A.	17.9	13.1 ± 2.3	5.0	21.8 ± 0.8
*ERBB4*	212812097	SNV	G		100.0	N.A.	72.3	N.A.	43.1	45.2 ± 3.7	5.1	26.8 ± 1.1
*FGFR3*	1807894	SNV	A		100.0	100.0	100.0	100.0	100.0	100.0 ± 0.0	100.0	100.0 ± 0.0
*FLT3*	28602367	SNV	A		49.5	N.A.	N.A.	N.A.	12.4	17.8 ± 0.8	0.0	N.A.
*FLT3*	28610183	SNV	C		100.0	64.3	100.0	65.2	82.4	81.1 ± 0.8	66.8	69.0 ± 0.9
*HRAS*	534242	SNV	C		98.9	47.8	38.9	48.5	58.5	60.6 ± 2.5	47.2	48.2 ± 2.9
*KDR*	55946354	SNV	A		47.9	N.A.	N.A.	N.A.	12.0	17.9 ± 1.2	0.0	N.A.
*KDR*	55972974	SNV	T		47.1	N.A.	N.A.	N.A.	11.8	16.8 ± 1.1	0.0	N.A.
*KRAS*	25398281	SNV	A		47.7	N.A.	N.A.	N.A.	11.9	12.1 ± 1.8	0.0	N.A.
*KRAS*	25398285	SNV	T		N.A.	100.0	N.A.	N.A.	25.0	36.6 ± 1.2	93.0	80.3 ± 1.4
*MET*	116339672	SNV	T		N.A.	70.3	N.A.	N.A.	17.6	19.2 ± 0.8	65.4	43.2 ± 1.1
*NOTCH1*	139390822	SNV	G		N.A.	100.0	N.A.	N.A.	25.0	33.4 ± 1.1	93.0	70.6 ± 1.5
*PDGFRA*	55141055	SNV	G		100.0	100.0	100.0	100.0	100.0	100.0 ± 0.0	100.0	100.0 ± 0.0
*PDGFRA*	55152040	SNV	T		N.A.	N.A.	51.3	N.A.	12.8	8.7 ± 0.2	3.6	18.1 ± 1.4
*PIK3CA*	178917005	SNV	G		N.A.	N.A.	100.0	N.A.	25.0	14.7 ± 0.9	7.0	28.0 ± 0.8
*PIK3CA*	178927410	SNV	G		N.A.	N.A.	47.1	N.A.	11.8	8.8 ± 0.0	3.3	13.5 ± 1.0
*PIK3CA*	178952085	SNV	G		47.7	N.A.	N.A.	N.A.	11.9	12.3 ± 1.0	0.0	N.A.
*PTEN*	89711881	SNV	G		N.A.	N.A.	N.A.	100.0	25.0	18.8 ± 1.9	0.0	N.A.
*RET*	43613843	SNV	T		100.0	67.5	100.0	N.A.	66.9	70.6 ± 2.8	69.8	76.2 ± 1.5
*RET*	43615612	SNV	G		49.1	N.A.	N.A.	N.A.	12.3	14.6 ± 2.4	0.0	N.A.
*RET*	43615633	SNV	G		N.A.	65.1	N.A.	N.A.	16.3	22.8 ± 0.1	60.5	44.9 ± 1.5
*SMAD4*	48586344	SNV	T		50.6	N.A.	N.A.	N.A.	12.7	15.9 ± 1.6	0.0	N.A.
*SMARCB1*	24176287	SNV	A		52.1	N.A.	46.3	N.A.	24.6	20.2 ± 0.6	3.2	15.6 ± 1.0
*SMO*	128846374	SNV	A		51.0	N.A.	N.A.	N.A.	12.8	12.7 ± 1.8	0.0	N.A.
*TP53*	7577120	SNV	A		N.A.	N.A.	100.0	N.A.	25.0	20.7 ± 0.8	7.0	32.8 ± 1.6
*TP53*	7577539	SNV	T		N.A.	99.9	N.A.	N.A.	25.0	27.6 ± 1.1	92.9	67.8 ± 1.4
*TP53*	7579472	SNV	G		84.2	N.A.	90.8	N.A.	43.8	57.6 ± 8.3	6.4	37.9 ± 5.2

N.A., Not Applicable; a, the MiaPaCa-2 cell line has a homozygous deletion of the *CDKN2A* gene

In terms of accuracy, we correlated the variant findings for the HCT116 and SK-MEL-28 cell lines analyzed in this study with the results obtained by the Genomics and Bioinformatics Group (GBG) from NCI, by querying the CellMiner database [18]. This database contains genomic information on the cell lines from the NCI-60 project. These cell lines have been intensely investigated, and a comprehensive analysis of coding variants in these cell lines have been identified by whole exome sequencing (WES). Thus, we found that all but two variants had previously been identified by WES. In the HCT116 cell line, two variants were not found on the CellMiner database: SMAD4_48586344_C > T and RET_43615612_A > G.

The variant in the *SMAD4* gene is located in an intronic region; therefore it may not have been detected by WES. In order to validate the presence of this variant in our cell line, we designed a multiplex allele-specific PCR (ASPCR) assay to assess the presence of such variant, which, according to our results, seemed to be found in our clone of HCT116 cells, in a heterozygous fashion. Primers were designed to co-amplify a conserved region of the *SMAD4* gene (286 bp), encompassing the C > T variant, and a variant-specific amplicon (181 bp) in the same reaction tube. Two PCR master-mixes were designed: one that would detect the variant, and another one that would detect the normal sequence in that position. Similarly, primers were designed to co-amplify a conserved region of the *RET* gene (268 bp), encompassing the A > G variant, and a variant-specific amplicon (176 bp) in the same reaction tube. As shown on Fig. 3, HCT116, but not the other cell lines, showed evidence of the variant, confirming our sequencing results.

**Fig. 3:** Multiplex ASPCR results. Novel variants found in the *SMAD4* and *RET* genes were confirmed by ASPCR and capillary electrophoresis using Lab-on-a-Chip technology performed on the 4 cell lines used in this study. For the *SMAD4* gene, the 286 bp peak corresponds to a conserved region encompassing the C > T variant at the 48,586,344 position in the hg19 reference genome and the 181 bp peak corresponds to the variant-specific amplicon. For the *RET* gene, the 268 bp peak corresponds to a conserved region encompassing the A > G variant at the 43,615,612 position in the hg19 reference genome, and the 176 bp peak corresponds to the variant-specific amplicon

In addition, we found 100 % agreement with the variants identified by our CHP2 assay in the well-characterized reference DNA sample NA12878 from the HapMap project [19] with those reported by others sequencing the same genomic regions (Life Technologies, Carlsbad, CA).

### Effect of formalin fixation and Laser Capture Microdissection (LCM)

In order to assess the potential effects of formalin fixation on variant identification, we sequenced DNA isolated from fresh-frozen cell lines and from DNA isolated from FFPE cell pellets prepared from the same cell lines. We then compared the variants identified in the fresh-frozen cell lines and their FFPE counterparts. Excellent Pearson’s correlations were observed for all the variant frequencies identified in each pair of samples (i.e. MIA-PaCa-2 *r* = 0.989, HCT116 *r* = 0.986, SK-MEL-28 *r* = 0.995, H1975 *r* = 0.992; p < 0.001).

In addition, we assessed the potential effects of Laser Capture Microdissection (LCM) on variant detection by sequencing DNA isolated from a whole tissue section from a NSCLC case, containing near 70 % neoplastic cells, and from DNA isolated from tumor cells enriched by LCM from the same case. We then compared the variants and their frequencies identified in each sample type. An excellent Pearson’s correlation (*r* = 0.909, *p* = 7.3 x 10^−8^) was observed between the two sample types, while Pathogenic/Likely Pathogenic somatic variants, such as *EGFR* NM_005228.3: c.2307_2308insGCCAGCGTG (p.Val769_Asp770insAlaSerVal) and *TP53* NM_000546.5: c.659A > G (p.Tyr220Cys) were over-represented (i.e. at higher allelic variant frequencies) in the LCM sample compared to the whole tissue sample, as expected.

### VariantCaller plugin parameters

The seven barcoded FFPE cell line mix samples with known variant frequencies were used to establish cutoff values for critical run and TVC parameters to achieve enough stringency (fewer false positives), while maintaining high sensitivity (fewer false negatives) in the variant calling process. Critical parameters, including those chosen to customize the TVC plugin, with their z and cutoff values, are listed in Table 4. Graphical representations of the Shapiro-Wilk normality test for three of the critical parameters are shown in Fig. 4. Thus, based on the normal distribution of the critical parameters, the established cutoff values were used as custom TVC plugin parameters, which were recorded in a JSON text format. The TVC Quality parameter failed to show a normal distribution, but the log_10_-transformed Quality values did. Thus, a log_10_-transformed cutoff value was calculated, instead.

**Table 4:** Cutoff values for Ion Torrent PGM sequencing and TVC parameters

	Mean	S.D.	Confidence Level	z	Cutoff (at z-score)
Coverage	1231	526	95 %	199	200
Number of ≥ Q20 bases	2.5E + 07	2.4E + 06	95 %	2.0E + 07	2.0E + 07
Quality (log_10_)	3.65	0.45	99 %	2.48	300^a^
Strand Bias	0.7	0.04	99 %	0.79	0.79

S.D., standard deviation; a, anti-logarithm of the found z value

**Fig. 4:** Normal quantile plots. The Shapiro-Wilk test was performed to assess the normality of the distribution of each of the adjustable parameters: coverage (**a**), ≥Q20 Bases (**b**), TVC Quality (**c**), and TVC Quality (Log_10_) (**d**). The expected quantile line for a normal distribution is shown in red

### Clinical specimens

After processing the previously tested 55 clinical specimens, we compared the *KRAS*, *BRAF* and *EGFR* variants obtained by NGS with our previous single gene assay results (Table 5). One clinical sample showed a L858R mutation in the *EGFR* gene using the single gene assay, which has a LoD of 1 % of mutant allelic frequency, in the context of normal DNA, but that variant was undetectable in the CHP2 assay. Upon visualizing the BAM file with the IGV tool, we found that the variant was present in < 4 % of the reads (Fig. 5), therefore below the LoD of the NGS-based assay. Thus, we found that the CHP2 assay performs with 96.7 % sensitivity and 100.0 % specificity for these three genes, when compared to single gene assays, which have a LoD of 1 % for *BRAF* and *EGFR*, and 5 % for *KRAS*.

**Table 5:** Clinical specimen results for known *KRAS*, *EGFR* and *BRAF* mutations

	*KRAS* or *EGFR* or *BRAF* Mutation Status	
Sample_ID	Single-Gene Assay	CHP2 Assay
DNA_01	*EGFR* c.2369C > T (p.Thr790Met)	*EGFR* c.2369C > T (p.Thr790Met)
DNA_02	*EGFR* c.2156G > C p.Gly719Ala	*EGFR* c.2156G > C p.Gly719Ala
DNA_03	Negative	Negative
DNA_04	Negative	Negative
DNA_05	*EGFR* Exon 20 INS	*EGFR* c.2307_2308ins9 (p.V769_D770insASV)
DNA_06	Negative	Negative
DNA_07	Negative	Negative
DNA_08	*EGFR* c.2369C > T (p.Thr790Met)	*EGFR* c.2369C > T (p.Thr790Met)
DNA_09	*EGFR* c.2369C > T (p.Thr790Met)	*EGFR* c.2369C > T (p.Thr790Met)
DNA_10	*EGFR* Exon 19 DEL	*EGFR* c.2236_2250del15 (p.E746_A750delELREA)
DNA_11	Negative	Negative
DNA_12	Negative	Negative
DNA_13	Negative	Negative
DNA_14	Negative	Negative
DNA_15	Negative	Negative
DNA_16	Negative	Negative
DNA_17	Negative	Negative
DNA_18	Negative	Negative
DNA_19	Negative	Negative
DNA_20	Negative	Negative
DNA_21	*KRAS* c.35G > T (p.Gly12Val)	*KRAS* c.35G > T (p.Gly12Val)
DNA_22	Negative	Negative
DNA_23	*EGFR* c.2582 T > A (p.Leu861Gln)	*EGFR* c.2582 T > A (p.Leu861Gln)
DNA_24	*EGFR* c.2582 T > A (p.Leu861Gln)	*EGFR* c.2582 T > A (p.Leu861Gln)
DNA_25	Negative	Negative
DNA_26	*BRAF* c.1799 T > A (p.Val600Glu)	*BRAF* c.1799 T > A (p.Val600Glu)
DNA_27	*KRAS* c.34G > A (p.Gly12Ser)	c.34G > A (p.Gly12Ser)
DNA_28	Negative	Negative
DNA_29	*EGFR* c.2155G > A (p.Gly719Ser)	*EGFR* c.2155G > A (p.Gly719Ser)
DNA_30	Negative	Negative
DNA_31	Negative	Negative
DNA_32	*KRAS* c.34G > T (p.Gly12Cys)	c.34G > T (p.Gly12Cys)
DNA_33	*BRAF* c.1798_1799delGTinsAA (p.Val600Lys)	*BRAF* c.1798_1799delGTinsAA (p.Val600Lys)
DNA_34	*BRAF* c.1798_1799delGTinsAA (p.Val600Lys)	*BRAF* c.1798_1799delGTinsAA (p.Val600Lys)
DNA_35	*EGFR* Exon 19 DEL	*EGFR* c.2235_2246del12 (p.Glu746_Glu749del)
DNA_36	Negative	Negative
DNA_37	*EGFR* c.2573 T > G (p.Leu858Arg)	*EGFR* c.2573 T > G (p.Leu858Arg)
DNA_38	*EGFR* c.2573 T > G (p.Leu858Arg)	*EGFR* c.2573 T > G (p.Leu858Arg)
DNA_39	*KRAS* c.34G > T (p.Gly12Cys)	c.34G > T (p.Gly12Cys)
DNA_40	Negative	Negative
DNA_41	*KRAS* c.38G > A (p.Gly13Asp)	c.38G > A (p.Gly13Asp)
DNA_42	*KRAS* c.38G > A (p.Gly13Asp)	c.38G > A (p.Gly13Asp)
DNA_43	*EGFR* c.2573 T > G (p.Leu858Arg)	Negative
DNA_44	*EGFR* Exon 20 INS	c.2312_2314dupACC (p.Pro772delinsHisPro)
DNA_45	Negative	Negative
DNA_46	Negative	Negative
DNA_47	*KRAS* c.35G > T (p.Gly12Val)	c.35G > T (p.Gly12Val)
DNA_48	Negative	Negative
DNA_49	Negative	Negative
DNA_50	*BRAF* c.1799 T > A (p.V600Glu)	c.1799 T > A (p.V600Glu)
DNA_51	*KRAS* c.35G > A (p.Gly12Asp)	c.35G > A (p.Gly12Asp)
DNA_52	*BRAF* c.1799 T > A (p.Val600Glu)	*BRAF* c.1799 T > A (p.Val600Glu)
DNA_53	*KRAS* c.35G > T (p.Gly12Val)	*KRAS* c.35G > T (p.Gly12Val)
DNA_54	*EGFR* c.2573 T > G (p.Leu858Arg)	*EGFR* c.2573 T > G (p.Leu858Arg)
DNA_55	*BRAF* c.1799 T > A (p.Val600Glu)	*BRAF* c.1799 T > A (p.Val600Glu)

**Fig. 5:** Visualization of the L858R *EGFR* mutation. The *EGFR* T > G variant indicated by the black arrow at the 55,259,515 position in the hg19 reference genome was present in a small number of reads and, therefore, was not called by the TVC

### Common variants and artifacts

From the variants found in the 55 archived clinical samples, the four cell lines and the reference DNA sample NA12878, we observed a number of recurrent variants that seem to be detected in the majority of the samples. A list of these common variants is shown in Table 6. Some of the variants correspond to sequencing artifacts, such as homopolymers [13]. Other variants seem to systematically occur at the end of an amplicon, and others seem to correspond to SNPs with a high global minor allele frequency (MAF) (e.g., rs1050171 [A/G], MAF A: 0.4183).

**Table 6:** List of common variants

Gene_Position_Variant	Class
EGFR_55249063_G > A	High Allele Frequency SNP
FGFR3_1807894_G > A	High Allele Frequency SNP
FLT3_28610183_T > C	High Allele Frequency SNP
PDGFRA_55141055_A > G	High Allele Frequency SNP
CSF1R_149433596_A > C	End of Amplicon
CSF1R_149433597_C > T	End of Amplicon
STK11_1220321_T > C	Homopolymer
PTEN_89711834_INS > T	Homopolymer
RB1_48953805_DEL > A	Homopolymer

### Performance of the Quality Control (QC) Material

We have developed and implemented a high quality and cost-effective control material for routine utilization in the CHP2 assay on FFPE samples. This QC material consists of a FFPE mixture of cell lines derived from pancreatic (MIA-PaCa-2), colon (HCT116), melanoma (SK-MEL28) and lung (H1975) cancer. This cell line mixture was created to assess 8 somatic variants, including 7 SNVs and 1 small DEL located in five different genes (*BRAF, EGFR, KRAS*, *PIK3CA*, and *CTNNB1*) at different allelic frequencies, and was subjected to formalin fixation and paraffin embedding to mimic routine FFPE clinical specimens. The performance characteristics of the QC material were established over 10 consecutive runs. Average reads on target for the QC material was 95.13 % ± 2.33 % and average uniformity on target areas was 98.26 % ± 0.68 %. During the initial 10 consecutive runs, all expected somatic variants in the QC material were consistently called at variant frequencies ranging from 9.1 % (CV = 11.1 %) to 37.9 % (CV = 2.8 %) (Table 7). Subsequently, for every batch/run, DNA isolated from a single 10-μm section of this cell mixture block was barcoded along with other six samples, and the allele frequencies for variants called on the five genes were recorded and plotted in Levey-Jennings charts for every clinical run (Fig. 6).

**Table 7:** Performance characteristics of the QC material

Gene Symbol	hg19 Coordinates	Variant Type	Variant	Mean Frequency (%)	Standard Deviation	%CV
*BRAF*	140453136	SNV	A	18.5	1.5	7.9 %
*EGFR*	55242487	SNV	T	17.1	1.4	7.9 %
*EGFR*	55249071	SNV	T	28.6	1.7	6.1 %
*EGFR*	55259515	SNV	G	23.4	1.5	6.5 %
*KRAS*	25398281	SNV	A	9.6	0.7	7.0 %
*KRAS*	25398285	SNV	T	37.9	1.1	2.8 %
*PIK3CA*	178952085	SNV	G	9.1	1.0	11.1 %
*CTNNB1*	41266134	DEL	CTT	11.5	2.0	17.8 %

**Fig. 6:** Continuous monitoring of the QC material using Levey-Jennings plots. The lowest frequency of a SNV (**a**) and of a small DEL (**b**) from the 8 variants detected in the QC material listed in Table 7 were monitored on each run over a period of 6 months using Levey-Jennings plots. The plots show the expected mean value, previously assessed by 10 independent runs, as well as expected limits: two standard deviations (SD) (*hatched lines*), and three SD (*solid lines*). All variants frequencies are within three standard deviations of the mean expected value

## Discussion

In the recent years, NGS has been mainly used in genomic-based research projects. The advent of cost-effective desktop instruments, such as the Illumina MiSeq and the Ion Torrent PGM, enabled the transition of NGS from genomic research into the clinical arena. In order for NGS technology to translate into clinical testing, it must meet the rigorous quality assurance and quality control protocols used in CLIA-certified laboratories and be used on a routine basis, replacing single-gene assays. This transition has already started, primarily for rare inherited disorders, including prenatal testing, and cancer theragnosis.

In this study, we assessed the performance characteristics of the Ion AmpliSeq™ Cancer Hotspot Panel v2 (CHP2) assay by sequencing well-characterized cell lines derived from pancreatic, colorectal, lung cancer, and melanoma, as well as different mixtures of fresh-frozen and FFPE DNA isolated from these cell lines. Thus, we assessed the sensitivity of the CHP2 assay in detecting low frequency somatic variants, or the assay’s limit of detection (LoD), as well as the assay’s precision and accuracy. In addition we evaluated the effects of sample barcoding, formalin fixation and paraffin embedding, as well as the impact of performing laser capture microdissection, on variant calling for these samples.

By establishing sequencing run quality control and variantCaller (TVC) cutoff parameters, we were able to customize the analysis pipeline for the CHP2 assay. Thus, we assessed the accuracy of the assay by sequencing 55 archival DNA samples, previously tested on single-gene mutational analysis assays, as well as one DNA sample from the HapMap project [19].

Overall, our results show that the CHP2 assay has a LoD of 4 % of allelic frequency when barcoding up to 7 fresh-frozen and FFPE-derived DNA samples in a single Ion 316™ chip, with good precision as shown by excellent repeatability (intra-run) and reproducibility (inter-run) metrics. Likewise, the CHP2 assay showed high accuracy when correlating the variants found on DNA isolated from the HCT116 and SK-MEL-28 cell lines, which have been previously analyzed by WES by the Genomics and Bioinformatics Group (GBG) from NCI [18]. Thus, we found that 19 out of the 21 variants had previously been identified by the NCI’s GBG. The two unconfirmed variants seen in our laboratory were further identified by ASPCR assays, confirming that these two variants might be specific to the cell lines grown in our laboratory, and not a sequencing artifact. Moreover, we found an excellent correlation with previously reported variants and their frequencies for the well-characterized reference DNA sample NA12878 from the HapMap project [19]. The fact that all-21 variants found in the SK-MEL-28 and HCT116 DNA samples by the CHP2 assay were confirmed by WES by the GBG from NCI, or by ASPCR as presented here, allows us to confidently report somatic variants detected in clinical specimens, when all the QC criteria presented in this study are met in the clinical run. This is in line with a recently published study that concludes that confirmatory analysis by Sanger sequencing of variants detected by NGS testing that meets appropriate quality thresholds is “unnecessarily redundant” [23].

Furthermore, when sequencing previously tested 55 clinical specimens, we found that the CHP2 assay performs with 96.7 % sensitivity and 100.0 % specificity for the *KRAS*, *BRAF* and *EGFR* genes, when compared to single gene assays results, using as little as 1–10 ng of FFPE DNA as template. In addition, we have identified common variants that were called in the majority of the samples, and we were able to ascertain that they correspond to either sequencing artifacts or to SNPs with a high global MAF. Thus, we were able to flag these common variant in our analysis pipeline, to not include them in the final report.

It has been recommended that, in order to assure the quality of this, or any NGS-based assay in routine clinical laboratory practice, efforts should be made to establish a suitable and robust reference or control material, and the sequence of such control material could be used to monitor quality as the technology and/or the analysis pipeline evolve. Such a control material should be well characterized and have similar variants as those targeted by the assay, and should include SNVs and Indels. These variants may be pathogenic or not, and should be located in genomic regions targeted by the assay [24].

Therefore, we developed and tested a quality control (QC) material by mixing, fixing and embedding the four cell lines used in the assay validation process. The performance characteristics of this control were assessed during 10 independent consecutive runs and mean and ranges were established to monitor each clinical run thereafter. The fact that the QC material was created on a patient-like matrix (i.e., FFPE cell block) makes it an excellent quality control material to monitor every step of the assay, from DNA extraction to data analysis pipeline and variant calling. Also, since a single 10-μm section is used in each batch of samples for a run, the costs of running this QC material are dramatically lower than those of running some commercially available materials. Moreover, the robust performance characteristics of such QC material ensures the generation of high quality sequence data from NGS testing of FFPE specimens, even close to the limit of detection of the assay. It is worth noting that, even though we have shown that we are able to consistently call variants at low frequencies, near 9 %, in the QC material presented here, this alone does not ensure that variants at lower frequencies (i.e. <9 %) will be confidently called by the assay in every run. A thorough analytical validation, specifically well-designed experiments to assess the LoD of the assay, is required to ensure that low frequency variants are reliably called by targeted NGS assays for somatic testing of FFPE specimens.

## Conclusions

In summary, during the validation process of the CHP2 assay, we have been able to customize the analysis pipeline, including the variant calling process, resulting in a highly sensitive, precise and accurate clinical assay. Moreover, we successfully developed a robust QC material that ensures consistent patient results in every clinical run. Even more importantly, this QC material, with a relative low manufacturing cost, has been instrumental to assess the performance of the CHP2 assay after each instrument preventive maintenance service, as well as minor software upgrades, which are prone to occur frequently in this rapidly evolving field.
